# Elucidation of the Key Therapeutic Targets and Potential Mechanisms of Marmesine against Knee Osteoarthritis via Network Pharmacological Analysis and Molecular Docking

**DOI:** 10.1155/2022/8303493

**Published:** 2022-12-12

**Authors:** Hanbing Song, Hongpeng Liu, Xiaodong Li, Bing Lv, Zonghan Tang, Qipeng Chen, Danqi Zhang, Fei Wang

**Affiliations:** Heilongjiang University of Traditional Chinese Medicine, Harbin, 150000 Heilongjiang Province, China

## Abstract

**Background:**

Marmesine, a major active ingredient isolated from *Radix Angelicae biseratae* (Duhuo), has been reported to have multiple pharmacological activities. However, its therapeutic effects against knee osteoarthritis (OA) remain poorly investigated. The present study is aimed at uncovering the core targets and signaling pathways of marmesine against osteoarthritis using a combined method of bioinformatics and network pharmacology.

**Methods:**

We utilized SwissTargetPrediction and PharmMapper to collect the potential targets of marmesine. OA-related differentially expressed genes (DEGs) were identified from GSE98918 dataset. Then, the intersection genes between DEGs and candidate genes of marmesine were subjected to protein-protein interaction (PPI) network construction and functional enrichment analysis. The core targets were verified using the molecular docking technology.

**Results:**

A total of 320 marmesine-related genes and 5649 DEGs and 60 ingredient-disease targets between them were identified. The results of functional enrichment analyses revealed that response to oxygen levels, neuroinflammatory response, PI3K-Akt signaling pathway, MAPK signaling pathway, FoxO signaling pathway, and osteoclast differentiation was identified as the potential mechanisms of marmesine against OA. EGFR, CASP3, MMP9, PPARG, and MAPK1 served as hub genes regulated by marmesine in the treatment of OA, and the molecular docking further verified the results.

**Conclusion:**

Marmesine exerts the therapeutic effects against OA through multitarget and multipathways, in which EGFR, CASP3, MMP9, PPARG, and MAPK1 might be hub genes. Our research indicated that the combination of bioinformatics and network pharmacology could serve as an effective approach for investigating the potential mechanisms of natural product.

## 1. Introduction

Knee osteoarthritis (OA) is a common chronic osteoarthropathy that is characterized by joint space stenosis, bone hyperplasia, cartilage degeneration, and synovitis [1]. Knee dysfunction, chronic pain, malformation, and stiffness of the joint are the major clinical manifestations of OA. Besides, approximately 18% of women and 9.6% of men over 60 years suffered from OA [2]. Disability and chronic pain associated with OA could cause suicidal emotions, depression, and anxiety [3]. At present, the surgery, exercise, intra-articular injection, and oral drug therapy are the major therapies of OA. However, these treatments remain limited [4, 5]. Thus, it is necessary to develop a novel and effective therapy with less systemic toxicity and better bioavailability.

Chinese herbal medicine is the most commonly complementary and alternative medicine for OA treatment in China [6–8]. Many active natural products could be used as substitutes and valuable sources of anti-OA drugs, which might be worthy of further study. *Radix Angelicae biseratae* (Duhuo) is the root of the *Angelica biserrata* and has long been used to treat inflammation and arthralgia syndrome by alleviating pain and eliminating dampness [9]. Over 53 chemical ingredients have been identified from *Radix Angelicae biseratae*; of these volatile oil and coumarins are the primary constituents. However, the active ingredient of *Radix Angelicae biseratae* is complex, and the key active ingredient remains unknown. Marmesine is a furanocoumarin compound isolated from *Radix Angelicae biseratae*. It also has been reported to exhibit multiple pharmacological activities, including anticancer, antiangiogenic, anti-inflammatory, and hepatoprotective effects [10–13]. However, the therapeutic effects and potential mechanism in the treatment of OA remain poorly investigated.

Because natural products have multiple targets and exhibit a wide range of pharmacological effects, it is a great challenge to understand the corresponding biological functions and pathways of hub molecular targets. Network pharmacology is a novel and efficient tool to systematically uncover all potential targets, functions, and mechanisms of active ingredients at the system and molecular levels. It also provides a systematic and holistic perspective for analyzing drug activities [14]. In the present study, we combined bioinformatics and network pharmacology approaches to identify the potential targets and mechanisms of marmesine against OA. This study is aimed at uncovering the multitarget and multipathway of marmesine in the treatment of OA and providing the scientific basis for the prevention and treatment of OA.

## 2. Materials and Methods

### 2.1. Identification of OA-Related Genes

We downloaded the transcriptome profiles of OA patients (GSE98918 dataset) from the GEO database (https://www.ncbi.nlm.nih.gov/). Then, we used the robust multiarray average method to carry out data standardization preprocessing. The limma package of R software was applied to identify the differentially expressed genes (DEGs) between healthy samples (*n* = 12) and OA samples (*n* = 12), and the cut-off criteria were set as follows: *p* value < 0.05 and ∣logFC | ≥0.3 [15]. The volcano map of genes was visualized by ggplot2 package of R software. The heat map of top 20 genes was visualized by ComplexHeatmap package of R software.

### 2.2. Collection of Potential Targets

First, the 2D chemical structure of marmesine was downloaded from the PubChem database (https://pubchem.ncbi.nlm.nih.gov/). SwissTargetPrediction is a web server that aims to predict the potential targets of small molecules based on a combination of 2D and 3D similarity measures with known ligands [16]. PharmMapper is a web server to predict target candidates for the small molecules by pharmacophore mapping approach [17]. Then, we used the SwissTargetPrediction and PharmMapper databases to collect the potential genes of marmesine [18, 19].

### 2.3. Construction of the Protein-Protein Interaction (PPI) Network

The overlapped genes associated with OA and marmesine were identified as candidate targets by the Venn tool. Then, these candidate targets were introduced into the STRING database (https://cn.string-db.org/), the species was chosen as Homo sapiens, and a required confidence score > 0.4 was set to generate the TSV format file [20]. PPI network was visualized by the Cytoscape software (3.8.0) [21]. The hub target was identified using the CytoNCA plugin of the Cytoscape software. We also used MCODE plugin of the Cytoscape software to generate the clusters. The “compound-target-pathway” network of OA was constructed using the Cytoscape software (3.8.0).

### 2.4. Enrichment Analysis of the Intersection Genes

To further investigate the potential mechanisms of marmesine in the treatment of OA, the clusterProfiler package and Bioconductor package of R software were applied to carry out the functional enrichment analysis on the intersection genes. A *p* value < 0.05 was used as the cutoff criterion.

### 2.5. Molecular Docking

The hub target crystal structure was downloaded from the RCSB Protein Data Bank (https://www.rcsb.org/), of which the 3D protein conformations with a crystal resolution of smaller than 3 Å were selected. Then, the AutoDockTools 1.5.6 software was used to remove water, separate proteins, add nonpolar hydrogen, charge calculation, and construct the docking grid box. We used the AutoDock Vina 1.1.2 software to perform docking simulation, and the results were visualized via the PyMOL software.

## 3. Results

### 3.1. Identification of DEGs in OA Patients

Principal component analysis (PCA) was performed to assess the intragroup data repeatability, and the results showed that the repeatability of GSE98918 dataset is good (Figure 1(a)). As shown in Figure 1(b), a total of 5649 DEGs, including 3263 upregulated genes and 2386 downregulated genes, were identified through comparing 12 control samples and 12 OA samples. The heat map exhibited the top 20 genes with the most significant downregulation and upregulation (Figure 1(c)).

### 3.2. Collection of Target Genes of Marmesine and Intersection with Marmesine- and OA-Related Genes

The 2D chemical structure of marmesine is presented in Figure 2(a). SwissTargetPrediction and PharmMapper databases were used to collect the pharmacological targets of marmesine. After deletion of duplicate genes, we obtained 320 marmesine-associated genes (Figure 2(b)). Finally, 60 intersection genes of marmesine against OA were obtained via an overlap of OA-related genes with marmesine-related genes (Figure 3(a)). Among these overlapped genes, 29 were significantly upregulated and 31 were significantly downregulated (Figures 3(b) and 3(c)). These 60 overlapping genes were imported to the STRING database. Then, the PPI network was constructed, which contains 60 nodes and 154 edges (Figure 3(d)). This finding revealed the major interaction between marmesine and OA disease.

### 3.3. GO-BP and KEGG Enrichment Analyses

These 60 overlapping genes were further analyzed by enrichment analyses, which showed that marmesine impacted a series of GO-BP, such as cell growth, cellular response to external stimulus, response to oxygen levels, cellular response to environmental stimulus, positive regulation of growth, response to mechanical stimulus, heart growth, and neuroinflammatory response (Figures 4(a) and 5). Based on the KEGG enrichment results, the potential mechanisms of marmesine in the treatment of OA are mainly involved in the proteoglycans in cancer, PI3K-Akt signaling pathway, microRNAs in cancer, MAPK signaling pathway, FoxO signaling pathway, Ras signaling pathway, HIF-1 signaling pathway, endocrine resistance, osteoclast differentiation, ErbB signaling pathway, and EGFR tyrosine kinase inhibitor signaling pathway (Figures 4(b) and 5).

Furthermore, a component-target-pathway interaction network diagram was constructed via the Cytoscape software to further elaborate the relationship between the potential targets and corresponding pathways of marmesine against OA. As shown in Figure 6, the 60 red circular nodes represent the potential targets, the 8 light blue triangular nodes represent the KEGG pathways, the three light red dovetails represent the GO-BP pathways, and the green square node represents marmesine. The pathview package was applied to draw the pathway map of marmesine against OA, and the primary pathways were integrated to construct the pathway maps (Figures 7 and 8). These findings indicated that marmesine could take effect in OA treatment via multitargets and multipathways.

### 3.4. Construction of PPI Network and Identification of Hub Genes

The Cytoscape software was applied to construct the PPI network. Nine genes that were not linked to others in the network will be filtered out, including ARHGAP1, GSTA3, CRABP2, F11, BDKRB1, TPI1, CD1A, ITPKA, and ADAM33, and the PPI network contained 51 nodes and 154 edges (Figure 9(a)). Furthermore, the PPI network was divided into two modules using a MCODE plugin of the Cytoscape software. Meanwhile, the module 1 contains EGFR, CASP3, MMP9, PPARG, MAPK1, IGF1, KDR, RPS6KB1, MAPK8, CASP1, and ANXA5 (Figure 9(b)); the module 2 contains TYMS, CDK6, PLK1, and AURKA (Figure 9(c)). Then, CytoNCA plugin of the Cytoscape software was used to calculate the topological parameters of nodes based on degree, betweenness, and closeness. And top 5 genes (EGFR, CASP3, MMP9, PPARG, and MAPK1) were identified as hub genes and further validated using molecular docking analysis (Table 1).

### 3.5. Molecular Docking Results

A binding energy lower than -5 kcal/mol shows that bioactive compound had good binding ability with targets [22].  Figure 10 exhibits the major binding site between the amino acid residues of target protein and marmesine. Based on our molecular docking results, marmesine could bind well with target proteins (EGFR, CASP3, MMP9, PPARG, and MAPK1), among which MAPK1 exhibits the best binding effect (Table 2). Our findings indirectly revealed that the results of molecular docking are consistent with the network pharmacology results, which confirmed the screening results of network pharmacology.

## 4. Discussion

OA is a severe osteoarthropathy that impacts the whole joint system and often accompanied by the occurrence and development of synovitis [23]. Due to the complex pathological mechanism of OA, the specific pathogenesis has not been fully understood. Therefore, novel methods or drugs should be developed to prevent and treat OA. Chinese herbal medicine is the most commonly complementary and alternative medicine for OA treatment due to its multitarget and multipathway characteristics [6, 24]. *Radix Angelicae biseratae* (Duhuo) has long been used to treat arthralgia syndrome. Marmesine is the primary active component of *Radix Angelicae biseratae*, which has been reported to exert anti-inflammatory effect. However, the therapeutic effects and potential mechanisms of marmesine against OA have not been reported. Bioinformatics could identify new drug targets and predict the reposition of these licensed drugs in the treatment of additional indications [25]. Network pharmacology could well assess the overall relationship between diseases and drugs and has been widely used to establish guiding pharmacologic methods [26]. Therefore, we made a combination of bioinformatics and network pharmacology that might promote a further understanding of the pathogenesis of OA and identify the potential therapeutic targets of marmesine.

In the present study, 320 potential targets of marmesine and 5649 DEGs of OA were obtained. 60 cotargets were identified as the therapeutic targets of marmesine in the treatment of OA. Among them, six core targets (EGFR, CASP3, MMP9, PPARG, and MAPK1) were indicated to play an important role via CytoNCA plugin of the Cytoscape software. Furthermore, we performed the molecular docking analysis to further confirm the results of network pharmacology.

Epidermal growth factor receptor (EGFR) is a tyrosine kinase receptor, which plays an important role in the maintenance of superficial chondrocytes during the development of articular cartilage. It has been reported that chondrogenic EGFR signaling pathway involved in adult cartilage homeostasis and the progression of OA [27]. Previous study has demonstrated that mice with cartilage-specific EGFR deficiency promoted the progression of knee OA, and targeting EGFR signaling could effectively improve surgery-induced OA cartilage damage [28]. Furthermore, it has been reported that EGFR exerted a protective role during the development of OA via regulation of cartilage degradation [29]. Caspase-3 (CASP3) is an important member of the cysteine-aspartyl family with a vital role in apoptosis [30]. The expression and activation of CASP3 in the monocytes, macrophages, and synovium of rheumatoid arthritis patients were measured, and treatment with the CASP3 inhibitor could effectively improve arthritis symptoms [31]. Recent study has reported that the CASP3 is a potential biomarker for OA prognosis in Egyptian donkeys [32]. Matrix metallopeptidase 9 (MMP9) has been involved in the pathological process of various diseases, including OA. The increased expression of MMP9 promoted the progression of diabetic OA via accelerating chondrocyte apoptosis and suppressing cartilage differentiation [33, 34]. MMP9 was upregulated in synovial fluid of patients with OA [35], and increased MMP9 protein level may be related to the pathogenesis of OA [36]. Recent study has demonstrated that MMP9 is a potential diagnostic marker for OA patients [37, 38]. Peroxisome proliferator-activated receptor gamma (PPARG) is a nuclear receptor and involved in insulin sensitivity and energy metabolism. A recent study demonstrated that genetic polymorphisms of PPARG might promote the risk of the Kashin-Beck disease via disturbing ECM homeostasis [39]. Mitogen-activated protein kinase 1 (MAPK1) is a subfamily of the MAPK family that regulated a variety of cellular activities. miR-320c suppressed articular chondrocyte proliferation and evoked apoptosis via targeting MAPK1 [40]. Thus, the above target genes may all play an important role in the occurrence and progression of OA and are potential therapeutic targets for marmesine in the treatment of OA.

The enrichment analysis of these cotargets revealed that cellular metabolism, immune, and inflammatory pathways may be the potential mechanisms of marmesine in the treatment of OA. The representative pathways included PI3K-Akt signaling pathway, MAPK signaling pathway, FoxO signaling pathway, Ras signaling pathway, HIF-1 signaling pathway, osteoclast differentiation, ErbB signaling pathway, and EGFR tyrosine kinase inhibitor signaling pathway. MAPK signaling pathway is associated with the pathogenesis of arthritis and related diseases, especially OA [41]. For example, kinsenoside improved OA via inactivation of MAPK/NF-*κ*B signaling pathways [42]. Wang-Bi tablet could effectively suppress inflammatory response and articular cartilage damage via the downregulation of p38-MAPK and NF-*κ*B signal pathways [43]. Osteoclast differentiation plays an important role in the occurrence and development of temporomandibular joint OA [44]. For example, dihydroartemisinin could prevent osteoclast activation via inactivating NFATc1, MAPK, and NF-*κ*B pathways in a knee OA rat model [45]. IL-4 could inhibit osteoclast development and promote anti-inflammatory macrophages to protect against OA [46].

## 5. Conclusion

Our findings revealed that marmesine had multitargets and multipathways in the treatment of OA. Besides, EGFR, CASP3, MMP9, PPARG, and MAPK1 are the hub targets enriched in the MAPK signaling pathway and osteoclast differentiation and for marmesine to exert its anti-inflammatory and antiapoptosis effects against OA. Furthermore, molecular docking verification was performed to confirm that marmesine could form a stable docking model with these hub targets. Our research provides a systematic view of the potential therapeutic targets and signaling mechanisms of marmesine against OA based on network pharmacology and bioinformatics analyses, which may provide a novel therapeutic strategy for OA.

## Figures and Tables

**Figure 1:** Identification of DEGs in OA patients. (a) PCA for GSE98918 dataset. (b) Volcano diagram of DEGs in GSE98918 dataset. The blue dots represent the downregulated genes, and the red dots represent the upregulated genes. (c) Heat map of the top 20 genes with the most significant downregulation and upregulation in GSE98918 dataset. The purple group is the OA group, while the dark green group is the control group. The downregulated genes are exhibited in blue, and upregulated genes are showed in red.

**Figure 2:** Collection of marmesine-related genes. (a) The 2D chemical structure of marmesine. (b) The potential targets of marmesine.

**Figure 3:** Identification of the therapeutic targets of marmesine in the treatment of OA. (a) The intersection with marmesine- and OA-related genes. (b) Heat map of the 60 intersection genes in GSE98918 dataset. The purple group is the OA group, while the dark green group is the control group. The downregulated genes are exhibited in blue, and upregulated genes are showed in red. (c) Volcano diagram of 60 intersection genes in marmesine-related genes. The blue dots represent the downregulated genes, and the red dots represent the upregulated genes. (d) PPI network of 60 intersection genes.

**Figure 4:** Enrichment analysis of the 60 intersection genes. (a) Bubble diagram of the top 25 enriched biological process (BP). (b) Bubble diagram of the top 25 enriched Kyoto Encyclopedia of Genes and Genomes (KEGG) pathways. The colors of the bubble show the significance of enrichment, while size shows the gene count.

**Figure 5:** The representative pathways of marmesine in the treatment of OA. The results of representative pathways were presented by circle charts (a), circle plot (b), and chord plot (c).

**Figure 6:** The component-target-pathway network for marmesine. 60 red circular nodes represent the potential targets, the 8 light blue triangular nodes represent the KEGG pathways, the three light red dovetails represent the GO-BP pathways, and the green square node represents marmesine.

**Figure 7:** MAPK signaling pathway. The green and red rectangles indicate the potential targets of marmesine in the treatment of OA.

**Figure 8:** Osteoclast differentiation. The green and red rectangles indicate the potential targets of marmesine in the treatment of OA.

**Figure 9:** Construction of PPI network and identification of hub genes. (a) PPI network of potential targets of marmesine against OA. (b) Module 1 of PPI network (score: 9.6) (hub targets). (c) Module 2 of PPI network (score: 4). The color of nodes is proportional with the degree value, and the darker color indicates the greater value of nodes.

**Figure 10:** Molecular docking of marmesine with potential target proteins: EGFR (a), CASP3 (b), MMP9 (c), PPARG (d), and MAPK1 (e).

**Table 1:** Topological analysis of PPI network.

Target	Degree	Betweenness	Closeness
EGFR	23	585.6396	0.276243
CASP3	20	446.55685	0.276243
MMP9	18	226.11505	0.265957
PPARG	17	294.71487	0.263158
MAPK1	15	159.40509	0.261780

**Table 2:** Binding energies of marmesine to the hub target proteins.

Target proteins	Binding energy (kcal/mol)				
	EGFR	CASP3	MMP9	PPARG	MAPK1
Marmesine	-6.18	-6.3	-5.11	-5.35	-7.13

## Data Availability

All data that support the results of the present study are available from the corresponding authors upon request.
